This article has been retracted.

# Clinical Value of sTREM-1, PCT, and 1,3-*β*-D Glucan in Diagnosis of Immune-Associated Pulmonary Interstitial Disease with Fungal Infection

**DOI:** 10.1155/2022/6095441

**Published:** 2022-07-27

**Authors:** Lei Yan, Yuan Li, Chunye Wu, Yuquan Shi, Chunyu Kong

**Affiliations:** Department of Rheumatology and Immunology, Tianjin First Central Hospital, Tianjin 300192, China

## Abstract

**Background:**

Fungal infection in the lungs can cause fungal infectious diseases. This disease develops rapidly and involves a wide range. Pathogenic fungi are also more serious types of pathogenic bacteria. If it invades deep organs and tissues, it will endanger life, so it needs timely diagnosis.

**Aim:**

To investigate the diagnostic value of serum soluble myeloid cell triggering receptor-1 (sTREM-1), procalcitonin (PCT), and 1,3-*β*-D glucan detection in immune related lung disease complicated with fungal infection.

**Methods:**

In this study, a case-control study was conducted. 50 patients with immune-related pulmonary disease complicated with fungal infection (infection group) diagnosed by sputum culture in our hospital from January 2017 to December 2021 were selected as the control group, and 50 patients with immune-related pulmonary disease without fungal infection were selected as the control group. The levels of sTREM-1, PCT, and 1,3-*β*-D glucan were compared in the two groups. The receiver operating characteristic (ROC) was used to analyze the value of the three indicators in the diagnosis of immune-related pulmonary disease complicated with fungal infection, and the changes of the three indicators before and after treatment were compared.

**Results:**

The levels of sTREM-1, PCT, and 1,3-*β*-D glucan in the infection group were higher than those in the control group (*P* < 0.05). The levels of sTREM-1, PCT, and 1,3-*β*-D glucan in the infection group after treatment were significantly lower than those before treatment (*P* < 0.05). The AUC value of sTREM-1 in the diagnosis of immune-related pulmonary diseases complicated with fungal infection was 0.980, the sensitivity was 97.11%, and the specificity was 83.06%. The AUC value of PCT in the diagnosis of immune-related pulmonary diseases complicated with fungal infection was 0.860, the sensitivity was 80.00%, and the specificity was 72.41%. The AUC value of 1,3-*β*-D glucan in the diagnosis of immune-related pulmonary diseases complicated with fungal infection was 0.993, the sensitivity was 98.74%, and the specificity was 99.16%. The levels of sTREM-1, PCT, and 1,3-*β*-D glucan in the infection group after treatment were considerably lower than those before treatment, and the difference was statistically significant (*P* < 0.05).

**Conclusion:**

The detection of sTREM-1, PCT, and 1,3-*β*-D glucan levels has high clinical value for the diagnosis of immune-related pulmonary diseases complicated with fungal infection.

## 1. Introduction

The main clinical features of immune-related lung diseases are alveolar wall thickening, inflammatory cell infiltration, and pulmonary interstitial fibrosis [1, 2]. Such patients have significantly reduced lung compliance, abnormal pulmonary ventilation function, and high mortality rate. Therefore, early diagnosis and treatment of immune-related lung diseases are needed to improve patients' quality of life [3, 4]. Patients need long-term use of antibiotics, but long-term use is prone to drug resistance, which is also a major cause of increased mortality. Pathogenic examination is often used to clarify the characteristics and drug resistance of secondary fungal infection in immune-related lung diseases. However, the error of this method is large, and there may be false positives, which requires more reliable diagnostic methods [5, 6]. Studies have shown that the ideal marker detection can judge the ability of fungal infection and distinguish the relationship between fungal infection and other infections. At present, serum soluble myeloid cell trigger receptor-1 (sTREM-l) and procalcitonin (PCT) are commonly used to evaluate the degree of some infectious diseases, but the specificity of these indicators is poor, which cannot accurately reflect the immune-related pulmonary interstitial disease with fungal infection [7, 8]. Studies have shown that [9] 1,3-*β*-D glucan is specifically expressed in fungal cell wall, and its abnormal expression can accurately reflect the degree of invasive pulmonary fungal infection. In addition, 1,3-*β*-D glucan is easier to identify the type of infection. At present, there are few studies on the combined detection of serum sTREM-1, PCT, and 1,3-*β*-D glucan in the diagnosis of immune-related pulmonary diseases complicated with fungal infection [10]. Based on the above background, this study explored the application value of 1,3-*β*-D glucan combined with conventional infection indicators in the diagnosis of immune-related pulmonary diseases complicated with fungal infections.

### 1.1. Core Tips

1,3-*β*-D glucan is specific to the fungal cell wall, and its level reflects the situation of pulmonary fungal infection. The two indicators of sTREM-1 and PCT are clinically recognized to identify the type and degree of fungal infection. At present, there are few studies on the combination of the above three indicators for the detection of immune-related lung diseases complicated with fungal infection. This study is to explore the above in order to find new diagnostic methods.

## 2. Materials and Methods

### 2.1. General Information

The study used a case-control study was conducted, and 50 patients with immune-related pulmonary disease complicated with fungal infection (infection group) diagnosed by sputum culture in our hospital from January 2017 to December 2021 were selected as the control group.

The following are the inclusion criteria: (1) diagnostic criteria for connective tissue diseases refer to CTD diagnostic criteria developed by the American College of Rheumatology [11] and patients with interstitial lung disease confirmed by high resolution CT (HRCT) examination. (2) Patients aged 18–79 years old. (3) The results of CT imaging and sputum culture were used as the gold standard for pulmonary fungal infection. The diagnostic criteria refer to the diagnostic criteria and therapeutic principles of invasive pulmonary fungal infection (draft) [12]. (4) There clinical manifestations of patients with fever, cough, expectoration, dyspnea, and poor effect of conventional antibiotic therapy. (5) The research programme was approved by the Medical Ethics Committee of our hospital and signed informed consent with the subjects. The following are the exclusion criteria: (1) chronic obstructive pulmonary disease and radiation pneumonitis, (2) severe heart failure (NYHA class ≥ II), (3) mental patients, (4) HIV infection, (5) use of immunomodulators in recent 1 month, and (6) organ transplant patients.

### 2.2. Indicator Detection Method

4 mlL of venous blood was collected and centrifuged at 3000 r/min for 15 min. Serum was separated and stored after centrifugation. ELISA was used to detect the levels of 1,3-*β*-D glucan, sTREM-1, and PCT. ELISA kit was purchased from RD Company of the United States and operated in strict accordance with the operating procedures. Firstly, 1,3-*β*-D glucan, sTREM-1, and PCT standards were prepared according to the requirements. The absorbance values of the standards at each concentration were detected by an enzyme-labeled instrument. The standard curve was drawn with the standard concentration as the abscissa and the absorbance value as the ordinate, and the linear relationship was recorded. Then each sample to be tested was configured as a specified concentration, and its absorbance value was measured under the same conditions. The absorbance value of each sample was substituted into the corresponding standard curve to obtain the concentration of each sample to be tested.

### 2.3. Fungal Susceptibility Test

Blood was collected from patients prior to antifungal therapy. Blood samples were also collected on the 7th and 14th days after treatment, and the samples were inoculated into Sapaul weak fungus medium and incubated in a constant temperature incubator for 24-48 h. If there is fungal growth in the weak medium of fungal Sabouraud, after aseptic processing, the species is identified on the VITEK2 automatic identification instrument. Then, it was judged by the Gram staining method. After gram staining was determined to be fungal infection, 3 mL of 0.45% saline was added to the test tube for culturing the fungus. Pure colonies were taken and added with an appropriate amount of distilled water to make their turbidity 0.5. Fungal ID plates were used to identify their typing, and vacuum-dropped bacterial liquid was taken to the drug sensitive plate. VITEK2 Compact automatic microbial analysis system was used to analyze the drug sensitive plate.

According to “Diagnostic Criteria and Therapeutic Principles of Pulmonary Fungal Infections” [13] to determine the type and results of infection, combined with the characteristics of the colony, the fluorescent staining results were observed under a high-power microscope: strong blue-green and weak blue-green are positive; no fluorescence or very weak fluorescence is negative.

### 2.4. Treatment Methods

Observation group: methylprednisolone, 8 ~ 24mg, twice a day; prednisone, 10 ~ 30mg, twice a day. After one month of continuous treatment, the dosage was gradually reduced until it was reduced to ≤10 mg/d. On this basis, the antifungal drugs selected included voriconazole, itraconazole, fluconazole, amphotericin B, and 5-fluorocytosine. The control group did not use antibiotics.

### 2.5. Statistical Processing

The sTREM-1, PCT, 1,3-*β*-D glucan, and other measurement indexes of the patients in this study were tested by normal distribution, and they were in line with the approximate normal distribution or normal distribution, using $\bar{x}\pm s$ to express. The *t* test was used for comparison between the two groups. The *χ*^2^ test was used for comparison between groups of enumeration data; the receiver operating curve (ROC) model was used for diagnostic analysis. Using professional SPSS21.0 software for data processing, test level *α* = 0.05.

## 3. Results

### 3.1. Comparison of General Data between the Two Groups

The basic data such as age, gender, BMI, smoking, drinking, and comorbidities of the two groups were compared (*P* > 0.05) (Table 1).

### 3.2. Comparison of Fungal Infection Types and Drug Resistance Types in 50 Patients in the Infection Group

The Fungal infection of fifty patients are mainly caused by aspergillus, Candida albicans, Candida krusei, Candida tropicalis, Candida glabrata, and Candida parapsilosis. It has certain resistance to amphotericin B, itraconazole, fluconazole, and voriconazole (Table 2).

### 3.3. The Levels of sTREM-1, PCT, and 1,3-*β*-D in the Two Groups Were Compared

The levels of sTREM-1, PCT, and 1,3-*β*-D glucan in patients with immune-associated pulmonary disease complicated with fungal infection (infection group) were higher than those in patients without infection (control group), and the difference was statistically significant (*P* < 0.05).  Table 3.

### 3.4. The Value of sTREM-1, PCT, and 1,3-*β*-D Glucan in the Diagnosis of Immune-Related Lung Diseases Complicated by Fungal Infection

The receiver operating characteristic (ROC) was plotted with pulmonary fungal infection as the dependent variable and sTREM-1, PCT, and 1,3-*β*-D glucan test results as independent variables. The AUC value of sTREM-1 in the diagnosis of immune-related pulmonary diseases complicated with fungal infection was 0.980. The AUC value of PCT in the diagnosis of immune-related pulmonary diseases complicated with fungal infection was 0.860. The AUC value of 1,3-*β*-D glucan in the diagnosis of immune-related pulmonary diseases complicated with fungal infection was 0.993. See Figure 1.

### 3.5. Comparison of sTREM-1, PCT, and 1,3-*β*-D Glucan Levels in Infection Group before and after Treatment

Patients in the infection group were treated with methylprednisolone combined with antibiotics. The average values of sTREM-1, PCT, and 1,3-*β*-D glucan after treatment were significantly lower than those before treatment, and the difference between the two groups was statistically significant (*P* < 0.05). (Table 4).

## 4. Discussion

In recent years, due to the extensive use of clinical immunosuppressants and chemotherapy drugs, the incidence of pulmonary fungal infection has gradually increased in clinical practice. Fungal infection has certain conditions, but it lacks characteristics and is difficult to diagnose, and the prognosis of patients is generally poor. Therefore, it is urgent to find more specific indicators in clinical practice, in order to improve the efficiency of diagnosis and guide clinical treatment [14].

According to previous studies [15], Candida albicans can be regarded as the main pathogen of fungal infection, and the infection rate of other pathogens has also been increasing due to the changing types of infection. The study results showed that Candida albicans, aspergillus, Candida krusei, Candida tropicalis, Candida glabrata, and Candida parapsilosis were the main pathogens of pulmonary fungal infection in immune-related lung diseases. For pathogenic infection, targeted anti-infective treatment should be given in a timely manner, and basic care should be strengthened to prevent the cross-infection. However, with the use of a large number of antibiotics, fungi developed resistence to some antifungal drugs, affecting the therapeutic effect. When more kinds of drugs are used, the infection rate of fungi will gradually increase. Clinically, there are significant differences in the sensitivity rate and drug resistance rate of different fungi to common antifungal drugs. Drug resistance monitoring in this study can provide guidance for clinical rational selection of therapeutic drugs.

This study results showed that the above pathogens had certain resistance to itraconazole, voriconazole, fluconazole, and amphotericin B. This is related to the difference in the selection of research subjects and also related to factors such as reduced immunity and long-term use of hormone drugs. Long-term use of drugs can cause more pathogenic bacteria in the lungs of patients; therefore, in the treatment of diagnosed patients and suspected patients, it is necessary to formulate anti-infective treatment plans as soon as possible, timely limit the development of the disease, and improve the patient's life rate [16]. In recent years, fungal drug resistance genes have been constantly changing, and there are also great differences in the selection of antifungal drugs, which also brings difficulties to the selection of clinical treatment drugs and methods [17].

sTREM-1 is easy to be detected, and abnormally high expression of TREM-1 can be found in the skin, lymph nodes, lung tissue, and alveolar macrophages in the inflammatory response of Gram bacteria and fungi. The study results showed that the levels of sTREM-1 and PCT in the infection group were considerably higher than those in the control group. The expression level of sTREM-1 was significantly increased under the action of bacteria. Similarly, fungi can also abnormally increase sTREM-1 levels. It is worth noting that Mycobacterium tuberculosis cannot increase sTREM-1 levels. The expression of sTREM-1 is specific to a certain extent, so it can reflect pulmonary fungal infection degree. sTREM-1 can reduce the expression of pro-inflammatory cytokines and play a protective role, but combined with the results of this study, its overexpression in infectious diseases will aggravate the degree of infection.

Under the normal physiological state of PCT, its level is relatively stable and will not be released into the blood, and its level in the peripheral blood is at a low level [18]. When microorganisms are infected, the body specifically expresses CALC-I, and the increase of its expression will increase the release of PCT. PCT also participates in the body's inflammatory response and is an important marker to measure the degree of the body's inflammatory response. Combined with the study results, the serum PCT level in patients with fungal infection was increased, and the positive rate of PCT was closely related to the degree of pulmonary infection. Previous studies have found that after local fungal infection in the lungs and digestive tract, the level of PCT increases significantly, and the level of PCT in fungal infections is also very high. The study results showed that the PCT levels of the patients in the infection group after treatment were significantly lower than those before treatment. The change of PCT level can help clinical evaluation of treatment effect, and the detection of sTREM-1 and PCT levels after treatment is helpful for clinical evaluation of treatment effect and adjustment of the dose of therapeutic drugs.

The study results showed that the level of 1,3-*β*-D glucan has expression specificity, which can reflect the degree of fungal infection of immune-related lung diseases and evaluate the therapeutic effect. This study combined the diagnostic sensitivity. When the fungus invades blood or tissues, after the digestion of phagocytes, a large amount of 1,3-*β*-D glucan is released from the fungal cell wall and enters the blood circulation. In superficial fungal infection and fungal colonization, 1,3-*β*-D glucan is not released, and 1,3-*β*-D glucan can specifically activate coagulation factor G in limulus components, so 1,3-*β*-D glucan can theoretically become an important detection method for the diagnosis of pulmonary fungal infection.

Previous studies have mostly studied the relationship between sTREM-1 and PCT levels and pulmonary fungal infection and found that their levels can reflect the degree of pulmonary fungal infection [19, 20]. A large number of studies have also confirmed that the serum level of 1,3-*β*-D glucan in patients with pulmonary fungal infection is increased, and the increase in the serum level of 1,3-*β*-D glucan in patients with fungal infection is more obvious than that in patients with bacterial infection. Detection of serum 1,3-*β*-D glucan in patients is helpful for early diagnosis of pulmonary fungal infection. It was reported that the levels of 1,3-*β*-D and sTREM-1 in the plasma of patients with pulmonary fungal infection increased. At present, there is no study on the combination of the above three indicators for the diagnosis of immune-related pulmonary diseases complicated with fungal infection. Based on the above background and research status, this study explored the significance of combined detection of sTREM-1, PCT, and 1,3-*β*-D glucan levels and obtained ideal results. In addition to joint detection, this study also studied the main pathogens and analyzed their drug susceptibility, which is of great significance for the diagnosis and treatment of diseases. Therefore, in the treatment of fungal infections secondary to immune-related lung diseases, antifungal drugs should be standardized and reasonably used to reduce the occurrence of drug resistance and further improve the quality of life of patients.

In summary, the detection of sTREM-1, PCT, and 1,3-*β*-D glucan levels has high clinical value for the diagnosis of immune-related pulmonary diseases complicated with fungal infection.

## Figures and Tables

**Figure 1:** ROC chart of sTREM-1, PCT, and 1,3-*β*-D glucan in the diagnosis of immune-related lung diseases complicated by fungal infection.

**Table 1:** General data comparison.

	Infection group (*n* = 50)	Control group (*n* = 50)	*t*/*χ*^2^	*P*
Age (years)	64.8 ± 7.1	66.1 ± 6.8	-0.935	0.352
BMI (kg/m^2^)	23.67 ± 1.83	24.03 ± 1.72	-1.014	0.313
Gender (%)			1.714	0.190
Male	32 (64)	38 (76)		
Female	18 (36)	12 (24)		
Smoking (%)			1.961	0.161
Yes	21 (42)	28 (56)		
No	29 (58)	22 (44)		
Drinking (%)			1.131	0.288
Yes	19 (38)	14 (28)		
No	31 (62)	36 (72)		
Concomitant disease (%)				
Hypertension	21 (42)	28 (56)	1.961	0.161
Diabetes	16 (32)	11 (22)	1.268	0.260
Coronary heart disease	6 (12)	3 (6)	1.099	0.295
Hyperlipidemia	19 (38)	23 (46)	0.657	0.418

**Table 2:** Comparison of fungal infection types and drug resistance types in 50 patients in infection group.

Fungus type	*n*	Itraconazole		Voriconazole		Fluconazole		Amphotericin B	
		Number of resistant strains	Resistance rate (%)	Number of resistant strains	Resistance rate (%)	Resistance rate (%)	Number of resistant strains	Number of resistant strains	Resistance rate (%)
Aspergillus	16	4	25.00%	6	37.50%	12	75.00%	4	25.00%
Candida albicans	9	1	11.11%	2	22.22%	4	44.44%	2	22.22%
Candida glabrata	6	1	16.67%	1	16.67%	2	33.33%	1	16.67%
Candida krusei	8	1	12.50%	2	25.00%	3	37.50%	1	12.50%
Candida tropicalis	6	0	0.00%	0	0.00%	3	50.00%	3	50.00%
Candida parapsilosis	5	0	0.00%	1	20.00%	2	40.00%	1	20.00%

**Table 3:** Comparison of the levels of sTREM-1, PCT, and 1,3-*β*-D glucan between the infection group and the control group ($\bar{x}\pm s$).

Group	n	sTREM-1 (ng/L)	PCT (ng/L)	1,3-*β*-D dextran (pg/mL)
Infection group	50	54.19 ± 9.57	577.4 ± 97.4	43.57 ± 14.84
Control group	50	33.20 ± 5.58	448.1 ± 56.0	8.30 ± 3.13
*t*		13.398	8.138	16.444
*P*		<0.01	<0.01	<0.01

**Table 4:** Comparison of sTREM-1, PCT, and 1,3-*β*-D glucan levels before and after treatment ($\bar{x}\pm s$).

Time	*n*	sTREM-1 (ng/L)	PCT (ng/L)	1,3-*β*-D dextran (pg/mL)
Before therapy	50	54.19 ± 9.57	577.4 ± 97.4	43.57 ± 8.84
After treatment	50	39.66 ± 7.40	483.5 ± 66.1	22.50 ± 5.58
*t*		8.493	5.641	14.252
*p*		<0.01	<0.01	<0.01

## Data Availability

No data were used to support this study.
